This article has been retracted.

# Clinical Efficacy and Safety Study of Mifepristone with Misoprostol Treatment in Patients with Missed Abortion

**DOI:** 10.1155/2021/9983023

**Published:** 2021-09-28

**Authors:** Xiaoying Zhao, Congyi Zhang, Haitao Lou, Chunfang Wu

**Affiliations:** ^1^Department of Pharmacy, Zhuji Maternal and Child Health Hospital, Zhuji, Zhejiang 311800, China; ^2^Department of Gynaecology, Zhuji Maternal and Child Health Hospital, Zhuji, Zhejiang 311800, China; ^3^Department of Traditional Chinese Medicine, Zhuji Maternal and Child Health Hospital, Zhuji, Zhejiang 311800, China

## Abstract

Currently, medication abortion is widely used in clinical practice in China. The aim of this study was to investigate the effect of mifepristone with misoprostol treatment on the efficacy of patients with missed abortion (MA) and the safety of this drug regimen. 95 patients with MA treated in our hospital from February 2019 to April 2021 were collected as the subjects of this study, and the patients were divided into the control and the research groups according to different treatment modalities. Among them, 46 cases in the control group were treated by diethylstilbestrol combined with oxytocin and 49 cases in the research group were treated by mifepristone combined with misoprostol, and both groups underwent curettage after medication. The rates of complete abortion, time of embryo expulsion, time of operation, intraoperative bleeding, time of postoperative vaginal bleeding, amount of vaginal bleeding, rate of one-time curettage, the levels of serum estradiol (E2), progesterone (P), *β*-chorionic gonadotropin (*β*-hCG), and interleukin-18 (IL-18), and the incidence of adverse effects in the two groups were examined and compared. Alanine transaminase (ALT), aspartate aminotransferase (AST), blood urea nitrogen (BUN), and serum creatinine (Scr) were used as indicators to evaluate the safety of the drug. The results showed that the rates of complete abortion and one-time curettage were significantly higher in the study group than in the control group, while the time of embryo expulsion, operation time, intraoperative bleeding, postoperative vaginal bleeding time, and vaginal bleeding were significantly lower than in the control group. The serum E2, P, and *β*-hCG levels before curettage in both groups were significantly higher, and IL-18 levels were significantly lower than those at the time of admission, with E2, P, and *β*-hCG levels increasing more and IL-18 levels decreasing more in the research group. After drug treatment, no abnormal changes in liver and kidney functions were observed in both groups, and the incidence of adverse reactions was at a similar and lower level in both groups. This shows that mifepristone with misoprostol is a safer and more effective drug regimen for the treatment of MA, which can regulate the levels of serum sex hormones and inflammatory factors in the body, promote the shedding of placental tissue, and create conditions for improving the rate of curettage.

## 1. Introduction

Missed abortion (MA) is a special case of spontaneous abortion in which an embryo or a dead fetus is retained in the uterus and cannot be expelled in time [1]. The incidence of MA in China has been on the rise in recent years due to factors such as rising life stress and deterioration of living environment [2]. Clearance is the main treatment for MA, but the death of the embryo absorbs a large amount of amniotic fluid causing organization of the tissue, and the necrotic tissues may form a tight connection with the uterine wall and cannot be completely detached from the uterine wall, which can lead to difficulty in scraping or hemorrhage after the scraping procedure [3]. If the pregnancy tissue remains in the uterine cavity for a longer period of time, it can also lead to tissue lysis and release of large amounts of hemolysin into the blood circulation of the pregnant woman, causing a coagulation disorder, which can cause massive uterine bleeding and even lead to diffuse intravascular coagulation [4]. Therefore, the use of medications or other treatments to promote the release of mechanized placental tissue from the uterine wall prior to cleansing surgery becomes crucial in the treatment of MA.

Current clinical management methods related to MA have been reported both domestically and abroad [5, 6]. Most of the patients were treated with estrogen drugs combined with uterine clearance in the past, but some of them could not achieve satisfactory cervical dilatation, which then led to incomplete clearance and seriously affected the quality of life of the patients after surgery. Along with the improvement of the clinical medication level, the clinical management protocol of MA has been improved in recent years. Mifepristone is a progesterone receptor antagonist with antiendometrial proliferation, menopause, and ovulation inhibition, which is widely used in the clinical myoma uterus and dysfunctional uterine bleeding [7]. Misoprostol, which is a derivative of prostaglandins, can cause the destruction of decidua and villus tissue and promote their exfoliation, as well as trigger the tightening of uterine smooth muscle. It can also soften the cervix to facilitate embryo expulsion by inhibiting the synthesis of collagen fibers [8].

In this study, we conducted a comparative analysis of the effects of enestrel combined with uterotonin therapy and mifepristone combined with misoprostol therapy on the clinical outcomes of MA patients and the drug safety of the different treatment regimens.

## 2. Information and Methods

### 2.1. Case Selection

#### 2.1.1. Case Source and Baseline Information

95 patients with MA, aged 21–40 years, with a mean age of 28.08 ± 6.27 years, who received treatment in our hospital from February 2019 to April 2021 were selected. The gestational weeks ranged from 8 to 12 weeks, with a mean of 10.26 ± 1.87 weeks. The number of pregnancies ranged from 1 to 4, with a mean of 2.13 ± 0.31. The number of deliveries was 0–2, with a mean of 0.62 ± 0.09. The duration of vaginal bleeding ranged from 1 to 17 days, with a mean of 12.52 ± 2.77 days. Among all patients, 27 had a history of miscarriage and 42 had previous vaginal deliveries (Table 1). 95 patients were randomly divided into the control group of 46 patients treated by diethylstilbestrol combined with oxytocin and the research group of 49 patients treated by mifepristone combined with misoprostol. Baseline data such as mean age, gestational week, number of pregnancies, number of deliveries, duration of vaginal bleeding, and number of previous miscarriages and vaginal deliveries were statistically analyzed between the control group and the research group, and the differences were not statistically significant (*P* > 0.05) and were comparable.

#### 2.1.2. Diagnostic Criteria [9]

(1) Disappearance of early pregnancy reaction and the patient has symptoms of preterm abortion or does not show any symptoms, (2) cervical opening in a closed state on gynecological examination, uterus smaller than the week of menopause, soft or medium texture, (3) positive urine pregnancy test result, and (4) dynamic ultrasound observation to determine intrauterine pregnancy, withered or stopped development of the gestational sac.

#### 2.1.3. Inclusion Criteria

(1) Meet the diagnostic criteria of MA, (2) aged 21–40 years old, (3) intrauterine pregnancy, (4) menopause stopped for less than 12 weeks, (5) no abnormalities in liver and kidney function tests at admission, and (6) filling out the informed consent form for this experiment and agreeing to join this experiment.

#### 2.1.4. Exclusion Criteria

(1) Patients with contraindications to the use of the drug in question. (2) Patients with a history of allergy to mifepristone or other drugs or who are allergic. (3) Patients who are hobby smokers and alcoholics. (4) Patients who have been taking prostaglandin inhibitors for a long time.

### 2.2. Methods

#### 2.2.1. Sources and Specifications of Drugs, Reagents, and Instruments

1. Drugs: mifepristone tablets (Shanghai Xinhualian Pharmaceutical Co., Ltd., approval number: H20000628, specification: 10 mg), misoprostol tablets (Shanghai Xinhualian Pharmaceutical Co., Ltd., approval number: H20094136, specification: 0.2 mg), diethylstilbestrol tablets (Guangdong Huanan Pharmaceutical Group Co., Ltd., approval number: H44024916, specification: 1 mg), and oxytocin injection (Guangzhou Baiyunshan Mingxing Pharmaceutical Co., Ltd., approval number: H44025245, specification: 1 ml: 5 units).
2. Reagents: serum estradiol (E2), progesterone (P), *β*-chorionic gonadotropin (*β*-hCG) determination kit (chemiluminescence method) (Beckman Coulter, USA), interleukin-18 (IL-18) ELISA kit (Shanghai Yubo Biotechnology Co., Ltd., China).
3. Instrument: VITROS 350 fully automatic biochemical analyzer (Orlando Clinical Diagnostics (USA) Co., Ltd.,).

#### 2.2.2. Treatment Methods

1. The control group was treated with diethylstilbestrol combined with oxytocin. Patients were instructed to take diethylstilbestrol tablets orally at a frequency of 1 mg each time, 3 times a day for 3 days. On day 4, an intravenous drip of oxytocin was administered, and curettage was performed on the same day.
2. Patients in the research group were treated with mifepristone combined with misoprostol in a sequential manner. Patients were instructed to fast for 2 hours before administration, and mifepristone tablets were taken once at 9:00 a.m. and once at 9:00 p.m. on day 1, day 2, and day 3, respectively, with 50 mg each time. 0.6 mg of misoprostol tablets were taken on an empty stomach after waking up in the morning on day 4, and curettage was performed after the embryonic tissue was expelled or vaginal bleeding.

#### 2.2.3. Observation Indexes

1. The time of embryo expulsion, operation time, intraoperative bleeding, one-time curettage rate, and postoperative vaginal bleeding were observed and recorded in both groups, and the results were compared. The adverse reactions, including nausea and vomiting, abdominal pain, and weakness, which occurred during the treatment, were recorded in both groups, and the total incidence was calculated and compared.
2. Laboratory index: on admission and before curettage, 5 mL of fasting venous blood was collected from patients in the early morning, and the serum was separated by centrifugation and placed in a refrigerator at −80°C for testing. The serum levels of E2, P, *β*-hCG, and IL-18 were measured by the immunochemiluminescence assay and IL-18 by the enzyme-linked immunosorbent assay (ELISA). The relevant steps were completed according to the kit instructions. The levels of alanine transaminase (ALT), aspartate aminotransferase (AST), blood urea nitrogen (BUN), and serum creatinine (Scr) were measured by a fully automatic biochemical analyzer as safety observation indexes.

#### 2.2.4. Evaluation of the Efficacy of Medication Abortion [10]

Patients were followed up regularly after the operation to observe the changes of vaginal bleeding and other symptoms, and the patients were evaluated at 3 levels of complete abortion, partial abortion, and invalid according to the changes of symptoms after medication and ultrasound examination results. Complete abortion: the patient's embryo sac was completely expelled within 48 h after the administration of the drug, and the ultrasound examination showed no intrauterine residue, vaginal bleeding lasted ≤7 days, no need for uterine evacuation, and the symptoms were completely eliminated. Partial miscarriage: the embryo sac was completely expelled within 48 h after dosing, ultrasound examination showed intrauterine residue less than 1 cm, and vaginal bleeding lasts for 15–27 days, requiring continued dosing or surgical intervention. Invalid: the embryo sac was still not expelled within 72 h after medication, and the embryo sac was found to be left in the uterine cavity by ultrasound examination, and aspiration was performed; or there was residue in the uterus by ultrasound examination during the follow-up consultation, and at the same time, excessive bleeding was observed and the uterus was cleared; or the embryo sac was expelled after medication, and vaginal bleeding lasts for more than 21 days and cleansing surgery was performed. Complete abortion rate = number of complete abortion cases/total cases × 100%.

### 2.3. Statistical Analysis Methods

The data of this study were organized and entered using Excel software, and the differences between the two groups were analyzed using SPSS 19.0 statistical analysis software, and graphs were made using Prism 8.0. The statistical data were expressed as (*n*, %), and the chi-square (*χ*^2^) was used; the measurement data were recorded as mean ± standard deviation ($\bar{x}$ ± *s*), and the *t*-test was performed after recording, and the test level of *P* < 0.05 was considered as a statistically significant difference.

## 3. Results

### 3.1. Comparison of the Efficacy of Medication Abortion

The efficacy of medication abortion in both groups was observed and counted at the end of follow-up, in which there were 29 patients with complete abortion (63.04%), 15 patients with partial abortion (32.61%), and 2 patients (4.35%) with ineffective medication in the control group; in the research group, there were 40 cases of complete abortion (81.63%), 8 cases of partial abortion (16.33%), and 1 case of ineffective (2.04%). The analyzed results showed that the rate of complete miscarriage was significantly higher in the research group than in the control group (*P* < 0.05, Figure 1).

### 3.2. Comparison of Intraoperative and Postoperative-Related Conditions

We observed and recorded the intraoperative and postoperative conditions of the two groups and compared them. The results of statistical analysis showed that the embryo expulsion time, operation time, intraoperative bleeding, postoperative vaginal bleeding time, and vaginal bleeding in the study group were significantly lower than those in the control group, and the rate of one-time curettage was significantly higher than that in the control group (*P* < 0.05, Figure 2).

### 3.3. Comparison of Serum E2, P, *β*-hCG, and IL-18 Levels at Different times

The results of each factor tested at the time of admission and before curettage in the two groups are as follows. At the time of admission, serum E2, P, *β*-hCG, and IL-18 were at similar levels in both groups, with no statistically significant differences (*P* > 0.05). Before curettage, serum E2, P, and *β*-hCG levels increased and serum IL-18 levels decreased in both groups compared with those at admission; compared with the control group, serum E2, P, and *β*-hCG levels were higher and serum IL-18 levels were lower in the study group before curettage (*P* < 0.05) (Figure 3).

### 3.4. Observation of Drug Safety

We used liver function and kidney function as the observation index of drug safety, and the test results are as follows. The levels of ALT, AST, BUN, and Scr were at similar levels in both groups from the time of admission to the time of clearing surgery, and there was no abnormal change in liver and kidney functions in both groups (*P* > 0.05, Figure 4), indicating that the safety of the treatment methods in both groups was good.

### 3.5. Comparison of the Incidence of Adverse Reactions

We observed and counted the adverse reactions in both groups, including nausea and vomiting, mild abdominal pain, and malaise, which were mild and showed a transient nature. In the control group, there were 2 cases of nausea and vomiting, 2 cases of mild abdominal pain, and 1 case of malaise, with an overall incidence of 10.87% (4/46). In the study group, nausea and vomiting occurred in 4 cases, mild abdominal pain in 3 cases, and malaise in 1 case, with an overall incidence of 16.30% (6/49). Comparison of the total incidence of adverse reactions in the two groups showed no statistically significant difference (*P* > 0.05, Figure 5).

## 4. Discussion

The occurrence of MA is associated with endocrine, intrauterine environment, poor dietary habits, immune deficiency, environment, and genetics and is a specific type of spontaneous abortion [11]. Curettage or medical abortion followed by curettage is the current mainstay of clinical treatment for MA, but direct curettage requires high technical requirements of the operator. Moreover, the retention of the embryo sac in the uterus can result in the organization of soft tissues and close adhesion with the uterine wall, increasing the difficulty of detaching both, which can often cause incomplete clearance and result in continuous vaginal bleeding or infection. Some patients even require multiple clearings, which carry a higher risk of complications and even secondary infertility [12, 13]. In this study, the combination of different drugs was used to treat MA patients, and the results showed that the time to embryo expulsion, duration of surgery, intraoperative bleeding, duration of vaginal bleeding, and bleeding volume were lower in the research group than in the control group, while the rate of complete abortion and primary curettage were significantly higher than in the control group. It is suggested that mifepristone and misoprostol can promote the shedding of organization tissues and uterine contractions and improve the efficiency of curettage.

Mifepristone is a new progesterone antagonist with high affinity, which binds to progesterone receptors and inhibits the progesterone from exerting its fetal preservation effect, and thus causes necrosis and shedding of the patient's decidua graviditatis and villi tissue [14]. In addition, it induces uterine contraction by releasing endogenous prostaglandins, which subsequently induce the detachment of the decidua from the uterine wall, softening and dilating the cervix to facilitate the expulsion of intrauterine tissue. As a steroidal structured progesterone receptor antagonist with a very high safety profile, mifepristone has no progestational, androgenic, estrogenic, or antiestrogenic activity and significantly improves the rate of complete abortions in patients [15, 16]. Misoprostol is a derivative of prostate E that exerts cervical softening and dilating effects by stimulating the release of various elastase enzymes from cervical fibrous tissue, and it also enhances uterine contraction [17]. The combination of the two can play a dual role of stripping embryonic tissue and dilating the cervix simultaneously.

Estrogen and progesterone play a key role in the establishment and continuation of pregnancy and the entire delivery process. P is the main biologically active progestin secreted by the ovary that binds to specific receptors in target tissues such as the endometrium and myometrium to maintain placental function [18]. It is also able to reduce the sensitivity of the uterine muscle to contraction to avoid abnormal uterine contractions during pregnancy [19]. E2 is an estrogen secreted by the placenta and ovaries, which can promote endometrial proliferation and lay the foundation for normal pregnancy, and its level in early pregnancy can reflect ovarian luteal function and the quality of the dominant follicle [20]. *β*-hCG is a glycoprotein hormone secreted by syncytial trophoblasts that can promote the secretion of estrogen and luteal growth to maintain normal pregnancy, and its level is positively correlated with trophoblast activity [21, 22]. Studies [23] proved that abnormalities in the function of the placenta, corpus luteum, and trophoblast cells often tend to affect their hormone secretion levels, thus leading to the development of MA. As a new type of chemotactic regulator with multiple biological activities, IL-18 can regulate the balance of T helper cell 1/T helper cell 2 (Th1/Th2) bidirectionally, and its overexpression can stimulate the increase of Th1 cells in cooperation with other inflammatory factors, shifting the Th1/Th2 balance toward Th1 and leading to the development of MA [24]. The results of this study showed that the level of *β*-hCG, P, and E2 was lower than conventional and the level of IL-18 was higher than conventional in the 2 groups at admission, indicating that MA patients had low estrogen and progesterone levels and were in a state of strong inflammatory response. The results of the preoperative tests showed a significant improvement of the abovementioned indicators in both groups, and the improvement was more obvious in the study group than in the control group, suggesting that mifepristone with misoprostol can promote the regulation of estrogen and progesterone and alleviate the inflammatory response of the body. In addition, the liver and kidney functions before and after treatment were normal in both groups; the incidence of adverse reactions was relatively low in both groups during the treatment period, and the adverse reactions that occurred were all transient, indicating that all the drugs in this study have a high safety level.

## 5. Conclusion

Mifepristone combined with misoprostol relieves inflammation in the organism, regulates serum and chorionic tissue sex hormone levels, promotes ablation of placental tissue, and sets the stage for successful curettage with a high degree of safety.

## Figures and Tables

**Figure 1:** Comparison of the efficacy of medication abortion. Compared with the control group, ^*∗*^*P* < 0.05.

**Figure 2:** Comparison of intraoperative and postoperative-related conditions. (a) Average embryo expulsion time. (b) Average operation time. (c) Mean intraoperative bleeding. (d) One-time curettage rate. (e) Average duration of vaginal bleeding. (f) Average vaginal bleeding volume. Compared with the control group, ^*∗*^*P* < 0.05.

**Figure 3:** Comparison of serum E2, P, *β*-hCG, and IL-18 levels at admission and before curettage. (a) Average serum E2 levels. (b) Average serum P levels. (c) Average serum *β*-hCG levels. (d) Average level of serum IL-18. Compared with the level of the same group at the time of admission, ^∧^*P* < 0.05; when compared with the control group, ^*∗*^*P* < 0.05.

**Figure 4:** Observation of drug safety. (a) Average level of ALT. (b) Average level of AST. (c) Average level of BUN. (d) Average level of Scr.

**Figure 5:** Comparison of the incidence of adverse reactions.

**Table 1:** Comparison of baseline data between the two groups.

Indicator	Control group (*n* = 46)	Research group (*n* = 49)	*P* value
Age (mean ± SD), years	27.96 ± 5.89	28.23 ± 6.42	0.832
Gestational week (mean ± SD), weeks	10.31 ± 1.86	10.18 ± 1.90	0.737
Pregnancy times (mean ± SD), times	2.10 ± 0.30	2.16 ± 0.32	0.349
Number of deliveries (mean ± SD), times	0.61 ± 0.08	0.63 ± 0.09	0.256
Vaginal bleeding time (mean ± SD), days	12.18 ± 2.59	12.74 ± 2.83	0.318
Miscarriage history (case, %)	12 (26.09%)	15 (30.61%)	0.625
History of vaginal delivery (case, %)	20 (43.48%)	22 (44.90%)	0.889

## Data Availability

The data used to support the findings of this study are available from the corresponding author upon request.
